This article has been retracted.

# Diagnostic Value of LH Peak Value of the GnRH Stimulation Test for Girls with Precocious Puberty and Its Correlation with Body Mass Index

**DOI:** 10.1155/2022/4118911

**Published:** 2022-06-02

**Authors:** Chunqing Zhao, Yulong Tang, Lirong Cheng

**Affiliations:** Department of Pediatrics, The Second People's Hospital of Nantong, Nantong, Jiangsu 226002, China

## Abstract

**Objective:**

To analyze the diagnostic value of luteinizing hormone (LH) peak value of the gonadotropin-releasing hormone (GnRH) stimulation test for girls with precocious puberty and its correlation with body mass index (BMI).

**Methods:**

A total of 230 girls with precocious puberty who came to our hospital for testing from June 2019 to June 2021 were selected and divided into a true group (*n* = 130) and sham group (*n* = 100) according to the results of the GnRH stimulation test. According to the BMI, the true group was further divided into a normal group (48 cases), overweight group (43 cases), and obese group (39 cases). The GnRH stimulation test was performed on all subjects, and the basal value and peak value of LH and the basal value and peak value of follicle-stimulating hormone (FSH) were recorded. The general data and serological indexes of the true group and the sham group were compared. Indicators of the GnRH stimulation test, breast stage, bone age, BMI, uterine volume, ovarian volume, and serological indicators (leptin, sex hormone-binding protein (SHBG), and adiponectin (APN)) were compared among the normal group, the overweight group, and the obese group.

**Results:**

There were no significant differences in age and breast stage between the true group and the sham group (*P* > 0.05). There were statistically significant differences in bone age, BMI, uterine volume, and ovarian volume between the two groups (*P* < 0.05). The LH base value, LH peak value, FSH base value, and FSH peak value in the true group were higher than those in the sham group, and the differences were statistically significant (*P* < 0.05). ROC curve analysis showed that the AUC of LH peak value in diagnosing girls with precocious puberty was 0.973, which was higher than 0.895, 0.875, and 0.912 of LH base value, FSH base value, and FSH peak value, respectively. There were statistically significant differences in LH base value, LH peak value, FSH base value, breast development stage, bone age, BMI, SHBG, leptin, and APN among the normal group, overweight group, and obese group (*P* < 0.05), but there were no significant differences in FSH peak value, uterine volume, and ovarian volume among the three groups (*P* > 0.05). There was a negative correlation between BMI, LH peak value, and FSH base value (*P* < 0.05), but there was no significant correlation between BMI and FSH peak value (*P* > 0.05).

**Conclusion:**

The LH peak value of the GnRH stimulation test has high diagnostic value for girls with precocious puberty, and BMI is negatively correlated with the LH peak value of CPP children.

## 1. Introduction

With the influence of dietary habits, modern industrial pollution, and other factors, the risk of precocious puberty in children increases [1]. Precocious puberty refers to the early onset of puberty, manifested as early secondary sexual characteristics and physical development, mainly in girls. Precocious puberty can be divided into central precocious puberty (CPP), peripheral precocious puberty(PPP), and partial precocious puberty (PT) according to whether the hypothalamic-pituitary-gonadal axis is activated or not [2]. True precocious puberty is the early initiation of the hypothalamic-pituitary-gonadal axis, and its process is similar to that of normal youth development. Under the central control, the hypothalamus releases gonadotropin-releasing hormone (GnRH) pulse to release LH secretion and stimulate gonadal development, which leads to the gradual development of the whole development process into fertile mature individuals. The peripheral precocious puberty of girls can be divided into homogenous precocious puberty and heterogenous precocious puberty (contradictory precocious puberty). Sexual precocity of same sex female points to the secondary sex characteristic that is female's secondary sex characteristic, sexual precocity of opposite sex. This points to a girl to appear male secondary sex characteristic, such as much hair, much acne, voice becomes low even clitoral hypertrophy to wait [3]. As the treatment and outcome of the two types are different, it is very important to distinguish them clinically early [4]. The gonadotropin-releasing hormone (GnRH) stimulation test is the gold standard for CPP diagnosis. Luteinizing hormone (LH) is a GnRH analogue, which interacts with follicle-stimulating hormone (FSH) to promote follicle maturation, stimulate estrogen secretion, and promote the production and maintenance of the luteum. HPGA mainly depends on the frequency and intensity of GnRH, LH, and FSH pulse release [5]. There is a close relationship between childhood obesity and precocious puberty, the accumulation of body fat will lead to the occurrence of precocious puberty, and a certain amount of fat storage is one of the main factors for the initiation of puberty. In addition, children with precocious puberty also have an obesity trend [6]. At the same time, other studies showed that body mass index (BMI) could affect the GnRH stimulation test, and the peak of LH stimulation was negatively correlated with BMI [7]. However, there are few studies on the impact of BMI on various indicators of the GnRH stimulation test in China. Based on this, this study is aimed at exploring the diagnostic value of LH peak value of the GnRH stimulation test for girls with precocious puberty and its correlation with BMI, in order to provide reference for the clinical diagnosis and treatment of girls with precocious puberty. The report is as follows.

## 2. Materials and Methods

### 2.1. Research Subjects

This study was a retrospective study. The girls with possible precocious puberty who came to our hospital for testing from June 2019 to June 2021 were selected and divided into the true group and sham group according to the GnRH stimulation test. Inclusion criteria for the true group were as follows: (1) subjects who meet the diagnostic criteria of CPP [8] and were confirmed after the GnRH stimulation test, with LH peak > 5.0 U/L and LH peak/FSH peak > 0.6; (2) bone age exceeding the actual age by 1 year or more; (3) pelvic B ultrasound showing gonadal development and uterine and ovarian body enlargement; (4) linear growth acceleration; and (5) complete case data and follow-up data. Exclusion criteria were as follows: (1) patients with a malignant tumor; (2) children with serious diseases such as heart, liver, and kidney diseases; (3) children complicated with uterine- or ovarian-related diseases; (4) precocious puberty caused by intracranial lesions or endocrine genetic diseases; (5) hormone therapy before admission; (6) presence of organic diseases such as those in the gonads, adrenal glands, hypothalamus, pituitary, and thyroid gland; (7) children with cognitive impairment or mental disorder; and (8) children lost to follow-up. Inclusion criteria for the sham group were as follow: (1) subjects who meet the diagnostic criteria of PPP [8] and had early breast development or pubic hair, without the development of other sexual characteristics; (2) bone age development being normal or less than one year older than actual; (3) the size of the uterus and ovary consistent with the actual age; (4) the LH peak value increase not obvious in the GnRH stimulation test; and (5) complete clinical data. Exclusion criteria were as follows: (1) patients with a malignant tumor; (2) children with serious diseases such as heart, liver, and kidney diseases; (3) organic diseases affecting the HPGA; (4) endocrine diseases, etc.; and (5) poor compliance. According to the cutoff value of BMI [9], the true group was divided into the normal group (48 cases) (BMI: 5%~), overweight group (43 cases) (BMI: 85%~), and obese group (39 cases) (BMI ≥ 95%). This study complies with the Declaration of Helsinki of the World Medical Congress.

Diagnostic criteria of CPP are as follows: according to guidelines by the Chinese Ministry of Health, central precocious puberty can be diagnosed if girls show signs of secondary sexual signs before the age of 8 years or have their first menstrual period under the age of 10 years with a growth surge and bone maturation. With the ultrasound examination standard, the ovary and uterus were enlarged, at least one ovarian volume is greater than 1 mL, and the follicle diameter is 4 mm. The diagnosis of CPP relies on the clinical presentation and the response of peak LH to GnRH stimulation trials. The truncation level for diagnostic CPP was at peak LH > 3.3 mIU/mL and LH/FSH > 0.6. Our article has passed the ethical approval by the hospital.

### 2.2. Methods

(1) General information of all subjects was collected, including age, height, weight, and medical history. BMI = weight (kg)/height^2^ (cm^2^), and sexual characteristics (breast stage, external genitalia, etc.) of children were detected. To distinguish breast tissue from adipose tissue, the girl's arms were raised during staging, and breast staging was evaluated by a professional pediatric endocrinologist using visual and palpation techniques. Staging was performed after evaluation by 2 specific pediatric endocrinologists to minimize error. Breast development was reconfirmed by ultrasound to distinguish real breast development from fat breast. (2) Bone age was measured by specialists of our hospital according to the GP atlas method [10] by taking frontal X-ray films of the left hand (including carpal bone and lower end of the radius and ulna). The ovarian and uterine volumes were measured by ultrasound (*V* = (*π*/6 × length × width × depth)), and the hypothalamic-pituitary gland was examined by MRI to exclude intracranial space-occupying lesions. (3) For the GnRH stimulation test, the serum LH and FSH were determined by immunochemiluminescence at 0, 30, 60, and 90 minutes after fasting injection with 2.5 *μ*g/kg gonadorelin (Maanshan Fengyuan Pharmaceutical Co., Ltd., SFDA approval number: H10960064, specification: 100 *μ*g) at 8~9 am. (4) For serological index detection, 3 mL of early morning venous blood was collected from children in the true group and centrifuged at 3000 r/min for 10 min, and the upper serum was absorbed and stored in the refrigerator at -80°C. Serum leptin was detected by the radioimmunoassay, the kit was purchased from Beijing North Biotechnology Co., Ltd., and the operation was carried out in strict accordance with the instructions. The electrochemiluminescence method was used to detect sex hormone-binding globulin (SHBG), the kit was purchased from Roche Diagnostics Co., Ltd., Germany, and the operation was carried out in strict accordance with the instructions. The adiponectin (APN) level was detected by ELISA, the kit was purchased from Zhejiang Huijia Biotechnology Co., Ltd., and the operation was carried out in strict accordance with the instructions.

### 2.3. Statistical Methods

SPSS 20.0 statistical software was used for statistical analysis, measurement data were expressed as $\bar{x}\pm s$, and the *t*-test was used for comparison of measurement data conforming to normal distribution and homogeneity of variance. Count data were expressed as rate (%), and the *χ*^2^ test was used for comparison. The diagnostic value of LH base value and peak value and FSH base value and peak value for girls with precocious puberty was analyzed by the ROC curve; the relationship between LH basal value, peak value, and FSH basal value, peak value, and BMI of the true group was analyzed by Pearson correlation; *P* < 0.05 was considered statistically significant.

## 3. Results

### 3.1. Comparison of General Data between the Two Groups

There was no significant difference in age and breast stage between the two groups (*P* > 0.05); there were statistically significant differences in bone age, BMI, uterine volume, and ovarian volume between the two groups (*P* < 0.05), as shown in Table 1.

### 3.2. Comparison of the Indicators of the GnRH Stimulation Test between the Two Groups

The LH base value, LH peak value, FSH base value, and FSH peak value of the true group were higher than those of the sham group, and the difference was statistically significant (*P* < 0.05), as shown in Table 2.

### 3.3. Diagnostic Value Analysis of Each Index of the GnRH Stimulation Test on Girls with Precocious Puberty

ROC curve analysis showed that the AUC of LH peak in diagnosing girls with precocious puberty was 0.973, which was higher than 0.895, 0.875, and 0.912 of LH base value, FSH base value, and FSH peak value, respectively, as shown in Table 3 and Figure 1.

### 3.4. Comparison of Each Index Level of the GnRH Stimulation Test in Patients with Different BMI in the True Group

There were statistically significant differences in LH base value, LH peak value, and FSH base value among the three groups (*P* < 0.05), and the LH base value, LH peak value, and FSH base value of the normal group were higher than those of the overweight and obese groups (*P* < 0.05), and the LH base value, LH peak value, and FSH base value in the overweight group were higher than those in the obese group (*P* < 0.05). There was no significant difference in FSH peak values among the three groups (*P* > 0.05), as shown in Table 4.

### 3.5. Comparison of Breast Development Stages, Uterine Volume, Ovarian Volume, and Bone Age in Patients with Different BMI in the True Group

There were significant differences in breast development stages and bone age among the three groups (*P* < 0.05), and the bone age of the normal group was lower than that of the overweight and obese groups (*P* < 0.05), and the bone age of the overweight group was lower than that of the obese group (*P* < 0.05); there was no significant difference in the uterine volume and ovarian volume among the three groups (*P* > 0.05), as shown in Table 5.

### 3.6. Comparison of Serological Indexes and BMI in Patients with Different BMI in the True Group

There were significant differences in BMI, SHBG, leptin, and APN among the three groups (*P* < 0.05), and the BMI and leptin of the normal group were lower than those of the overweight and obese groups (*P* < 0.05), while the BMI and leptin of the overweight group were lower than those of the obese group; the SHBG and APN in the normal group were higher than those in the overweight and obese groups (*P* < 0.05), and SHBG and APN in the overweight group were higher than those in the obese group (*P* < 0.05), as shown in Table 6.

### 3.7. Correlation Analysis between Each Index of the GnRH Stimulation Test and BMI in the True Group

BMI value was negatively correlated with LH base value, LH peak value, and FSH base value (*P* < 0.05), but there was no significant correlation between BMI and FSH peak value (*P* > 0.05), as shown in Table 7 and Figure 2.

## 4. Discussion

In recent years, with the development of society and the change of lifestyle, the daily intake of hormone-containing food and drugs by children has increased, resulting in an increased incidence of precocious puberty children [11]. Precocious puberty mainly refers to the development of secondary sexual characteristics before the age of 8 in girls and 9 in boys, among which the incidence of precocious puberty in girls is about 5 times that of boys, and precocious puberty children are prone to depression, inferiority complex, and other emotions, which affect their physical and mental health, resulting in an early closure of the epiphysis that makes the child's actual height lower than genetic expectations [12]. Precocious puberty is divided into CPP and PPP. CPP is caused by the premature initiation of HPGA, and its developmental process is consistent with the normal pubertal development sequence, but the age is advanced. CPP can lead to early epiphyseal healing due to advanced bone age, affecting the ultimate height of children [13]. PPP is characterized by the development of secondary sexual characteristics and increased levels of sex hormones without gonadal development [14]. Due to the different treatment methods and outcomes of the two types, early clinical identification is required.

The GnRH test is the gold standard for the diagnosis of CPP. Gonadotropin affects the normal growth and sexual development of children, and it is mainly controlled by GnRH. Under normal conditions, the female hypothalamus will release GnRH in a regular pulse mode after entering puberty, so that FSH and LH in blood show pulse fluctuations [15, 16]. However, HPGA is activated in children with CPP, leading to increased GnRH secretion and release of FSH and LH, which promotes menstruation and ovulation in children, resulting in accelerated growth and advanced bone age [17]. In this study, there were no significant differences in age and breast stage between the true group and the sham group, while there were differences in bone age, BMI, uterine volume, and ovarian volume between the two groups, suggesting that the uterus and ovaries of children in the true group began to develop and bone age was advanced. In general, the volume of the uterus and ovary varies little with age before puberty. Once puberty starts, the volume of the uterus and ovary increases significantly [18]. In the true group, under the stimulation of gonadotropin, gonadal development and secondary sexual characteristics appeared, and bone growth accelerated. At the same time, the LH base value, LH peak value, FSH base value, and FSH peak value of the true group were higher than those of the sham group, indicating that the sex hormone levels of the patients in the true group were higher than those in the sham group. Further ROC curve analysis found that the AUC of LH peak in diagnosing girls with precocious puberty was 0.973, which was higher than the 0.895, 0.875, and 0.912 of LH base value, FSH base value, and FSH peak value, respectively, suggesting that the LH peak value of the GnRH stimulation test has high diagnostic value in girls with precocious puberty.

Studies [19] have shown that precocious puberty is correlated with obesity, and obesity affects female hormone levels throughout preadolescence, adolescence, and adulthood. Other animal experiments [20] have shown that obesity caused by high fat diet is an important factor in inducing sexual maturity in mice. In this study, there were differences in breast development stage, bone age, LH base value, LH peak value, and FSH base value among the normal group, overweight group, and obese group. Further correlation analysis showed that BMI was negatively correlated with LH base value, LH peak value, and FSH base value, suggesting that obesity was related to breast development and bone growth in CPP children, and BMI was related to LH base value, LH peak value, and FSH base value to some extent. The low LH stimulation peak value in obese girls may be related to the existence of relatively high estrogen level and androgen level. High estrogen and androgen level can lead to decreased HPGA sensitivity and enhanced negative feedback inhibition, thus leading to the decrease in LH peak value [21]. This observation is consistent with the previous research. The mean LH and LH pulse amplitude and LH response to GnRH were decreased in obese women, and BMI was negatively correlated with LH pulse amplitude. Obese women had a significantly lower response to GnRH LH levels than the normal-weight group. These data are consistent with the possibility that obesity may have a subtle inhibitory effect on hypothalamic-pituitary-gonadal function in early adolescence [22, 23].

Obesity is also a state of insulin resistance. The increase in obesity-related insulin resistance leads to a decrease in SHBG synthesis in the liver, which leads to a decrease in estrogen inactivation [24]. This, in turn, allows unchallenged estrogen to remain in peripheral tissues for long periods of time. In addition, obesity-related hyperinsulinemia increases aromatase activity and promotes and accelerates the conversion of serum testosterone to estrogen [25]. Long-term high levels of estrogen help to reduce sensitivity and feedback inhibition of the hypothalamic-pituitary-gonad axis. These mechanisms lead to reduced LH levels in response to GnRH stimulation. The effect of obesity on LH secretion may also be related to leptin. Leptin is one of the several key signals that control food intake and energy balance and performs a variety of functions through central and peripheral receptors. Recent studies have found that exogenous adipokines, including leptin, cause alterations in GnRH pulse release by binding to leptin receptors in the hypothalamus [26]. APN is an important adipocytokine that participates in the regulation of sugar and fat metabolism and can increase insulin sensitivity. On the other hand, it is also affected by different levels of sex hormones. Studies have shown that high estrogen level can inhibit the secretion of APN [27]. In this study, there were significant differences in SHBG, leptin, and APN levels among the normal group, overweight group, and obese group, suggesting that obesity has a certain influence on the levels of SHBG, leptin, and APN and has a certain relationship with precocious puberty. The authors believe that the main reason is that the secretion of estrogen and androgen in girls with CPP increases significantly, and the accumulation of fat will cause compensatory hyperinsulinemia in girls, reduce the synthesis of SHBG, and affect the secretion of APN; at the same time, exogenous adipokine changes the release of GnRH pulse in the hypothalamus by binding with the leptin receptor, leading to the increase in LH and FSH levels [28, 29]. Therefore, obesity-induced changes in GnRH test results in girls with CPP may be related to the changes in SHBG, leptin, and APN levels, which suggests that the effect of BMI on the gonadal axis should be considered when interpreting GnRH test results. Of course, this study also has certain deficiencies. Due to the limitations of the sample size and selected groups, the study has certain limitations. Future studies will be conducted jointly with multiple centers to expand the sample size to ensure the accuracy and richness of this study.

In conclusion, the LH peak value of the GnRH stimulation test has high diagnostic value for girls with precocious puberty, and BMI is negatively correlated with the LH peak value of CPP children. Therefore, the influencing factors of BMI should be considered in the diagnosis of obese girls with CPP.

## Figures and Tables

**Figure 1:** ROC curve of the diagnostic value of each index of the GnRH stimulation test on girls with precocious puberty.

**Figure 2:** Correlation analysis between each index of the GnRH stimulation test and BMI in the true group.

**Table 1:** Comparison of general data between the two groups.

Factor	True group (*n* = 130)	Sham group (*n* = 100)	*Z*/*χ*^2^/*t*	*P*
Age (years)	7.44 ± 0.63	7.37 ± 0.59	0.859	0.392
Bone age	9.54 ± 1.04	8.05 ± 0.68	12.161	<0.001
BMI	17.68 ± 3.09	16.25 ± 3.33	3.363	0.001
Breast stage				
B2	67	56	0.790	0.374
B3	57	45		
B4	6	0		
Uterine volume (mL)	1.98 ± 0.52	0.82 ± 0.22	20.907	<0.001
Ovarian volume (mL)	2.15 ± 0.61	0.92 ± 0.26	18.880	<0.001

**Table 2:** Comparison of indicators of the GnRH stimulation test between the two groups ($\bar{x}\pm s$).

Group	Cases	LH (U/L)		FSH (mIU/mL)	
		Base value	Peak value	Base value	Peak value
True group	130	1.07 ± 0.50	11.97 ± 3.20	3.40 ± 1.03	14.21 ± 1.93
Sham group	100	0.44 ± 0.11	4.98 ± 1.84	2.06 ± 0.50	10.43 ± 2.58
*t*		12.366	19.498	11.966	112.712
*P*		<0.001	<0.001	<0.001	<0.001

**Table 3:** Diagnostic value analysis of each index of the GnRH stimulation test on girls with precocious puberty.

	AUC	*P* value	Cutoff value	95% confidence interval
LH base value	0.895	<0.001	0.69	0.853~0.937
LH peak value	0.973	<0.001	7.27	0.930~0.980
FSH base value	0.875	<0.001	2.53	0.833~0.918
FSH peak value	0.912	<0.001	12.65	0.871~0.953

**Table 4:** Comparison of each index level of the GnRH stimulation test in patients with different BMI in the true group ($\bar{x}\pm s$).

Group	Cases	LH (U/L)		FSH (mIU/mL)	
		Base value	Peak value	Base value	Peak value
Normal group	48	1.62 ± 0.27	14.50 ± 2.58	4.47 ± 0.50	14.24 ± 1.30
Overweight group	43	0.97 ± 0.15^①^	11.77 ± 2.39^①^	3.07 ± 0.71^①^	14.34 ± 1.69
Obese group	39	0.52 ± 0.14^①②^	9.10 ± 1.87^①②^	2.43 ± 0.46^①②^	14.02 ± 1.10
*F*		331.944	58.365	149.328	0.563
*P*		<0.001	<0.001	<0.001	0.571

^①^ *P* < 0.05 when compared with the normal group; ^②^*P* < 0.05 when compared with the overweight group.

**Table 5:** Comparison of breast development stages, uterine volume, ovarian volume, and bone age in patients with different BMI in the true group.

Group	Cases	Breast development stage			Uterine volume (mL)	Ovarian volume (mL)	Bone age (years)
		2	3	4			
Normal group	48	14	31	3	2.00 ± 0.59	2.19 ± 0.20	9.01 ± 0.93
Overweight group	43	16	26	1	1.90 ± 0.47	2.09 ± 0.53	9.49 ± 1.03^①^
Obese group	39	13	24	2	2.03 ± 0.44	2.17 ± 0.68	10.25 ± 0.74^①②^
*Z*/*t*		6.450			0.750	0.502	19.916
*P*		0.040			0.474	0.606	<0.001

^①^ *P* < 0.05 when compared with the normal group; ^②^*P* < 0.05 when compared with the overweight group.

**Table 6:** Related hormones and BMI in each group ($\bar{x}\pm s$).

Group	Cases	BMI	SHBG (mmol/L)	Leptin (ng/mL)	APN (ng/mL)
Normal group	48	15.08 ± 1.75	80.39 ± 10.32	5.02 ± 1.41	740.61 ± 114.85
Overweight group	43	17.33 ± 1.39^①^	63.21 ± 7.94^①^	11.60 ± 2.95^①^	644.51 ± 85.02^①^
Obese group	39	21.26 ± 2.18^①②^	46.33 ± 5.44^①②^	16.08 ± 2.62^①②^	471.08 ± 93.76^①②^
*F*		129.854	181.334	238.880	79.816
*P*		<0.001	<0.001	<0.001	<0.001

^①^ *P* < 0.05 when compared with the normal group; ^②^*P* < 0.05 when compared with the overweight group.

**Table 7:** Correlation analysis between each index of the GnRH stimulation test and BMI in the true group.

Related factors	BMI value	
	*r*	*P*
LH base value	-0.695	<0.001
LH peak value	-0.548	<0.001
FSH base value	-0.628	<0.001
FSH peak value	-0.059	0.507

## Data Availability

The labeled dataset used to support the findings of this study are available from the corresponding author upon request.
